# Absence of Cospeciation between the Uncultured *Frankia* Microsymbionts and the Disjunct Actinorhizal *Coriaria* Species

**DOI:** 10.1155/2014/924235

**Published:** 2014-04-22

**Authors:** Imen Nouioui, Faten Ghodhbane-Gtari, Maria P. Fernandez, Abdellatif Boudabous, Philippe Normand, Maher Gtari

**Affiliations:** ^1^Laboratoire Microorganismes et Biomolécules Actives, Université de Tunis El Manar (FST) et Université Carthage (INSAT), 2092 Tunis, Tunisia; ^2^Ecologie Microbienne, Centre National de la Recherche Scientifique UMR 5557, Université Lyon I, 69622 Villeurbanne Cedex, France; ^3^Laboratoire Microorganismes et Biomolécules Actives, Faculté des Sciences de Tunis, Campus Universitaire, 2092 Tunis, Tunisia

## Abstract

*Coriaria* is an actinorhizal plant that forms root nodules in symbiosis with nitrogen-fixing actinobacteria of the genus *Frankia*. This symbiotic association has drawn interest because of the disjunct geographical distribution of *Coriaria* in four separate areas of the world and in the context of evolutionary relationships between host plants and their uncultured microsymbionts. The evolution of *Frankia-Coriaria* symbioses was examined from a phylogenetic viewpoint using multiple genetic markers in both bacteria and host-plant partners. Total DNA extracted from root nodules collected from five species: *C. myrtifolia*, *C. arborea*, *C. nepalensis*, *C. japonica*, and *C. microphylla*, growing in the Mediterranean area (Morocco and France), New Zealand, Pakistan, Japan, and Mexico, respectively, was used to amplify glnA gene (glutamine synthetase), dnaA gene (chromosome replication initiator), and the nif DK IGS (intergenic spacer between nifD and nifK genes) in *Frankia* and the matK gene (chloroplast-encoded maturase K) and the intergenic transcribed spacers (18S rRNA-ITS1-5.8S rRNA-ITS2-28S rRNA) in *Coriaria* species. Phylogenetic reconstruction indicated that the radiations of *Frankia* strains and *Coriaria* species are not congruent. The lack of cospeciation between the two symbiotic partners may be explained by host shift at high taxonomic rank together with wind dispersal and/or survival in nonhost rhizosphere.

## 1. Introduction

The genus* Frankia* comprises nitrogen-fixing actinobacteria that are able to induce perennial root nodules on woody dicotyledonous plants called actinorhizals [1]. The actinorhizal plant families belong to three dicotyledonous orders: Fagales (Betulaceae,Casuarinaceae, and Myricaceae), Rosales (Elaeagnaceae, Rhamnaceae, and Rosaceae), and Cucurbitales (Coriariaceae and Datiscaceae) [2]. Analysis of the molecular phylogeny of members of* Frankia* genus consistently identifies four main clusters regardless of the typing locus used [3]. Three symbiotic* Frankia* clusters containing strains able to establish effective nodules and fulfill Koch's postulates and one atypical with strains unable to establish effective nodulation on their host plants have been defined among* Frankia* genera. Cluster 1 includes* Frankia* strains in association with Betulaceae, Myricaceae, and Casuarinaceae. Cluster 2 contains* Frankia* nodulating species from the Coriariaceae, Datiscaceae, and Rosaceae families as well as* Ceanothus* of the Rhamnaceae.* Frankia* strains in cluster 3 form effective root nodules on plants from members of the Myricaceae, Rhamnaceae, Elaeagnaceae, and* Gymnostoma* of the Casuarinaceae.

Symbiotic* Frankia* strains have been only isolated from Fagales (*Frankia* cluster 1) and the families Elaeagnaceae and Rhamnaceae (*Frankia* cluster 3) of the Rosales, while* Frankia* of cluster 2 have still not yet been isolated in culture despite repeated attempts [2]. The position in the* Frankia* phylogenetic tree of cluster 2 relative to the other clusters has varied depending on the marker used. It was proposed at the base using* gln*A and 16S rRNA genes [4, 5], derived with ITS 16S–23S rRNA genes [6] and concatenated* gyr*B,* nif*H and* gln*II genes [7] and should be clarified by the upcoming whole genome phylogeny. Nevertheless, a position at the base of all symbiotic lineages has been retained in the latest treatment of Bergey's manual [8].

Cross-inoculation studies using crushed nodules suggest that cluster 2 strains form a separate and unique host specificity group [9–11], even though provenances from the full geographical range have not yet been tested. Despite the high taxonomic diversity of host plants belonging to the cross-inoculation group of cluster 2 and its disjunct range, uncultured* Frankia* in root nodules of several host plants have so far shown a low level of diversity regardless of the typing locus used [6, 7, 11–16], suggesting a recent emergence, a strong and recent evolutionary bottleneck, or a nonrepresentative sampling. The time of emergence of all* Frankia* lineages is poorly documented as no convincing fossil remains. An equivalence between 16S rRNA sequences distance and time of emergence has been proposed by Ochman and Wilson [17] where 1% is equivalent to 50 million years, and since 4% divergence exists between* Frankia *cluster 2 and the other clusters, one would conclude that* Frankia* emerged 200  million years ago [5], which would mean that there is missing diversity either due to a recent evolutionary bottleneck or due to a lack of sampling [16]. A possibility thus exists that the missing variability in cluster 2 strains is due to the fact that sampling has so far been limited essentially to North American and Mediterranean areas.

Evidence for cospeciation has been found so far only in the case of* Casuarina* species growing in Australia and their* Frankia *[18] that are in their immense majority resistant to growth in pure culture. Among actinorhizal plants of the Cucurbitales subclade, the family Coriariaceae, with only one genus,* Coriaria*, contains about 17 species [19] that occur in four disjunct areas of the world: the Mediterranean, Southeast Asia, Central and South America, and the Pacific islands of New Zealand and Papua New Guinea [20–24]. Yokoyama et al. [19] considered that the Eurasian species are basal and have emerged some 60 million years ago. This date is in agreement with the 65 million years proposed by Bell et al. [25] based on multiple genes (*rbc*L, 18S rDNA,* atp*B) phylogeny, while the same authors propose an emergence of the Casuarinaceae at about 30 million years.

The present study was aimed at testing the hypothesis of cospeciation between uncultured* Frankia* microsymbionts and their* Coriaria* host species sampled from sites covering the full geographical range of the genus:* Coriaria myrtifolia* (Morocco and France),* C. nepalensis* (Pakistan),* C. arborea* (New Zealand),* C. japonica* (Japan), and* C. microphylla* (Mexico).

## 2. Materials and Methods

### 2.1. DNA Extraction, PCR Amplification, and Sequencing

Root nodules from naturally occurring* Coriaria* species (Table 1) were kindly provided by Dr. María Valdés (Escuela Nacional de Ciencias Biológicas, México, DF, México), Dr. Sajjad Mirza (National Institute for Biotechnology Genetic Engineering, Faisalabad, Pakistan), Dr. Warwick Silvester (University of Waikato, Waikato, New Zealand), Dr. Kawther Benbrahim (University of Fes, Fes, Morocco), Dr. Takashi Yamanaka (Forest and Forestry Products Research Institute, Ibaraki, Japan), and Dr. Jean-Claude Cleyet-Marel (INRA-IRD, Montpellier, France). Individual lobes were selected, surface-sterilized in 30% (vol/vol) H_2_O_2_, and rinsed several times with distilled sterile water. The DNA extraction from single nodule lobes was performed as previously described by Rouvier et al. [26]. Nodule lobes were crushed with sterile plastic mortars and pestles in 300 *μ*L of extraction buffer (100 mM Tris (pH 8), 20 mM EDTA, 1.4 M NaCl, 2% (wt/vol) CTAB (cetyltrimethyl ammonium bromide), and 1% (wt/vol) PVPP (polyvinyl polypyrrolidone)). The homogenates were incubated at 65°C for 60min, extracted with chloroform-isoamyl alcohol (24 : 1, vol/vol) and the resulting DNA was ethanol-precipitated and resolubilized. The extracted DNA was used for PCR amplification of both bacterial and plant DNA regions using the primers listed in Table 2. The amplicons were then cycle-sequenced in both directions using an ABI cycle sequencing kit (Applied Biosystem 3130). The nucleotide sequences obtained in this study were deposited in the NCBI nucleotide sequence database under the accession numbers given in Table 1.

### 2.2. Phylogenetic Analysis

*Frankia* strain CcI3 and* Casuarina equisetifolia* were used as outgroups in this study because they are physiologically distinct from the group studied yet phylogenetically close. The data sets were completed with homologous sequences present in the databases (Table 1). Alignments of* Frankia gln*A,* dna*A, and IGS* nif*D-K and* Coriaria mat*K and 18S rRNA-ITS1-5.8S rRNA-ITS2-28S rRNA were generated with ClustalW [27], manually edited with MEGA 5.0 [28]. Bacterial and plant sequences were separately concatenated and then used to examine maximum-likelihood cladogram evolutionary relationships of each symbiotic partner using 1000 bootstraps by following the GTR + G base substitution model. The distance between the sequences was calculated using Kimura's two-parameter model [29]. Phylogenetic trees were constructed using the Neighbor-Joining method [30] with 1000 bootstraps [31] as implemented in MEGA 5.0. In parallel, a Bayesian inference was realized with MrBayes [32] using the GTR + G model and 1,000,000 generations.

A statistical test for the presence of congruence between* Coriaria* and* Frankia* phylogenies was evaluated through global distance-based fitting in ParaFit program [33] as implemented in CopyCat [34] and tests of random association were performed with 9999 permutations globally across both phylogenies for each association.

An additional statistical test for correlation between geographical distances (obtained using http://www.daftlogic.com/projects-google-maps-distance-calculator.htm) and phylogenetic distances was made using Pearson's* r* correlation implemented in the R software [35].

## 3. Results

To avoid taxonomic ambiguities, DNAs from both* Coriaria* hosts and* Frankia* microsymbionts were characterized on the same root nodule tissues. The method of DNA isolation from root nodules used in this study yielded PCR-amplifiable DNA for both bacterial and plant PCR target sequences in all cases. However, in several instances it was easier to amplify* Frankia* than* Coriaria* DNA, which may have been mostly due to the specificity of the primer sets used. Thus, in this study, new primers were designed (Table 2).

For the bacterial microsymbionts, the average uncorrected* p*-distances (proportion of differences between sequences) were computed for each region and were found to be relatively small for* dna*A (*p* = 0.0378), intermediate for* gln*A (*p* = 0.0625), and high for IGS* nif*D-K region (*p* = 0.0833). Blast analyses of the individual genes permitted assigning them all to* Frankia* cluster 2. Nearly 3000 nucleotides were obtained by concatenating sequences of the three DNA regions.

Sequences variation for* Coriaria* species was small based on* mat*K gene (*p* = 0.0205) compared to ITS1-ITS2 sequences (*p* = 0.0423). By concatenating* mat*K and ITS1- ITS2 region, a composite sequence of 1500 nt was used for phylogenetic inference.

All studied sequences were analyzed independently to test for incongruence between the data sets for each symbiotic partner. Similar topologies have been generally observed between phylogenetic trees inferred from* gln*A,* dna*A, and IGS* nif*D-K sequences for* Frankia* and from* mat*K and ITS sequences for* Coriaria* regardless of the used phylogenetic methods (not shown).

The topologies of the trees obtained for the two symbiotic partners were not congruent (Figure 1). Moreover, global distance-based ParaFit analysis recovered mostly random associations between* Frankia* and* Coriaria* host plant species (*p* = 0.33) and rejected cospeciation hypothesis. On the microbial side, the New Zealand microsymbionts were at the root (Group A); then three groups emerged, group B comprising the Pakistani, Mexican, and Mediterranean symbionts from France, group C comprising microsymbionts from Morocco, and then group D comprising French and Japanese microsymbionts as well as the Dg1 reference sequence obtained initially from a Pakistani soil. On the host plant side, group 1 at the root comprises New Zealand and South American sequences, while group 2 comprises the Japanese, Mediterranean, and Pakistani sequences.

On the other hand, no significant correlations were found for* Frankia* symbionts (*r* ^2^ = 0.772; Fgeneticdist = (geogdist × 5.830E^−06^) + 2.541E^−02^) nor for the* Coriaria* host plants (*r* ^2^ = 0.883; Fgeneticdist = (geogdist × 2.023E^−06^) + 6.460E^−03^) (data not shown).

## 4. Discussion

Cospeciation has been postulated to have occurred in some* Frankia* actinorhizal host plants, in particular in the* Casuarina-Frankia* cluster 1b [18] but not in* Alnus-*infective and* Elaeagnus*-infective* Frankia* strains where many isolates able to fulfill Koch's postulates have been obtained. To test if cospeciation was general or an exception, it was decided to study uncultured* Frankia* microsymbionts and representative* Coriaria* hosts, a lineage where no* Frankia* isolate exists and where geographic discontinuities may have limited dispersion. DNA sequences were obtained from root nodules collected from New Zealand (*C. arborea*), Pakistan (*C. nepalensis*), Japan (*C. japonica*), Mexico (*C. microphylla*), and France and Morocco (*C. myrtifolia*) and multiple molecular markers were analyzed for phylogenetic inference.

Paleontological data based on macrofossils and pollen fossils have brought several authors [36–40] to conclude that the Coriariaceae had a Laurasian origin (North America and Eurasia). There have been a few dissenting opinions, in particular those of Croizat [41] and Schuster [42] who considered that* Coriaria *originated in Gondwana and migrated to the Northern Hemisphere. However, such paleontological studies are not very convincing, as it is recognizably hard to ascribe fossils to a given family and even more so to a given genus. Thus, several authors have been surprised by the results of molecular phylogeny positioning Coriariaceae close to the Datiscaceae. Molecular approaches would thus give support to a Gondwanan origin.

Yokoyama et al. [19] proposed that* Coriaria* species had emerged 59–63 million years ago, which is coherent with the date of 70 million years proposed by Bell et al. [25], considerably older than that proposed (30 million years) by the same authors for the Casuarinaceae.

Topology and clustering of* Coriaria* phylogeny obtained in the current study are similar to those obtained by Yokoyama et al. [19], while the position at the base of the host plant species from New Zealand,* C. arborea,* and the South American* C. ruscifolia* and* C*.* microphylla *species was contrary to that of Yokoyama et al. [19] who found the Eurasian species at the base using* rbc*L (a large subunit of ribulose 1,5-bisphosphate carboxylase/oxygenase) and* mat*K (maturase K) genes. The present study suggests that the* Coriaria *ancestor may have emerged between Asia and NZ and then dispersed worldwide and that the Asian lineage may have given rise relatively recently to the Mediterranean species, while the NZ lineage gave rise to the North American species (Figure 2).

Previous studies had concluded that* Frankia* cluster 2 had a low genetic diversity [6, 7, 16] but these studies had been focused on only part of the full diversity of the symbiotic* Coriaria-Frankia*, essentially in North America and Mediterranean. In this work we aimed to expand the scope of the study to the worldwide diversity and phylogeny of microsymbionts of* Coriaria* species. Four microbial subgroups were identified that did not fit to the geographic range of the host plants, while two host plant subgroups were identified. The position of subgroup A containing microsymbionts of New Zealand* C. arborea* at the base of* Frankia* cluster 2 is in agreement with previous study [16]. In view of previously reported data, members of cluster 2* Frankia* studied here were found to have relatively higher sequences variation (*p*-distance = 0.0625) than those reported by Vanden Heuvel et al. [16] (*p* = 0.00454) based on the same 460 nt of the* gln*A gene.

Molecular clock dating suggests that* Frankia* genus has emerged much earlier, 125 Myr bp before the appearance of angiosperm fossils in the Cretaceous period and the extant actinorhizal plants [4]. Normand et al. [5] using the 4% divergence in the 16S rRNA between cluster 2 and other* Frankia *lineages as equivalent to 50 MY/1% distance [17] concluded that the genus* Frankia* had emerged long before the extant dicotyledonous lineages. These authors proposed* Frankia* cluster 2 as the proto-*Frankia* as nonsymbiotic ancestor of 62–130 Myr bp [43] and 100–200 Myr bp [5]. Since the distance in the 16S rRNA gene between cluster 1a (*Frankia alni*) and cluster 1b is less than 1%, the date of emergence of the* Casuarina*-infective lineage has been proposed to be less than 50 million years [5]. Thus the* Casuarina*/*Frankia* 1b lineage is considerably younger than the* Coriaria*/*Frankia* lineage and would have had less time to migrate out of its cradle and mingle with other hosts in its new territories and lose the cospeciation signal.

Symbiotic partnership often tends to become obligatory, as in the case of* Casuarina* host plants, where* Frankia* is only present in soils close to the host plant [44], which means that the bacterium loses autonomy and becomes dependent on its host. Speciation of the host could then lead to synchronous speciation of its microsymbiont unless dispersal through long-distance carriers such as winds or migratory birds occurred or if there is survival of* Frankia* cluster 2 in the rhizosphere of nonhosts as was recently demonstrated for* Alnus glutinosa* in Tunisia [45]. The numerous transitions seen in the* Frankia* phylogenetic tree from one continent to another would reinforce the idea.

Yokoyama et al. [19] concluded from their study of the* Coriaria *species phylogeny that the Eurasian species had diverged earlier and are more diverse than other groups, but that nevertheless the origin of the genus could have been in North America, whence the South America and the Pacific species could have originated. Our study brings us to suggest a third possibility, Oceania, which could also be the origin of this actinorhizal symbiosis, which can be concluded from phylogenetic inferences positioning both bacterial and host plant partners as at the base to* Frankia*-Coriaria symbiosis. Another element that would support this hypothesis is the large number of extant species there; according to Yokoyama et al. [19] New Zealand would be home to 8 of the 17 existing species. A similar argument has often been made to establish Sub-Saharan Africa as the cradle of humankind [46] or Mexico for maize [47].

Comparison of both the plant and the microbe phylogenetic topologies did not show any evidence for cospeciation of* Frankia* microsymbiontsand their* Coriaria *host species. The results obtained in this study suggest that* Frankia* microsymbionts hosted currently by* Coriaria* species had probably dispersed globally as a proto-*Frankia*, a free living and nonsymbiotic ancestor. In parallel, the proto-*Coriaria *then diversified into the extant* Coriaria* species that appear to have been retreating given their scattered distribution, a trend possibly reinforced recently due to man uprooting because of the toxicity of the fruits for mammals [48, 49]. It can thus be hypothesized that* Coriaria* appeared in the Pacific Islands more than 70 million years ago and presumably was symbiotic from the start, before dispersing over all continents as they drifted apart. The* Coriaria *species diversified in their different biotopes, as they saw the appearance of other plants hosting the same microsymbiont of* Frankia *cluster 2 such as Datiscaceae*, Rosaceae, Ceanothus*, or even nonhost species such as* Alnus glutinosa* that was recently found to host* Frankia* cluster 2 in its rhizosphere [45]. Members of these alternative host plant species cooccur sympatrically with* Coriaria* such as* Ceanothus* and* Purshia* species in Mexico and* Datisca cannabina* in Pakistan. These* Frankia* cluster 2 host plant species have more extended geographic distribution and overlap in some instances* Coriaria*'s disjunct area and as a result can compensate* Frankia* microsymbionts remoteness, which would thus obscure the cospeciation signal. Cospeciation may also occur but subsequently is lost after bacterial mixing and fitness selection in the presence of “indigenous” and “dispersal” symbionts.

## Figures and Tables

**Figure 1:** Phylogenetic trees of the* Frankia* microsymbionts (left) and the* Coriaria* host plants (right). The* Frankia* tree was constructed using the* gln*A,* dna*A, and the* nif*D-K intergenic spacer, while the* Coriaria* tree was done using the* mat*K and the 18S rRNA-ITS1-5.8S rRNA-ITS2-28S rRNA with ML method using strain CcI3 and Casuarina as outgroups respectively for Frankia and hot plant phylogenetic trees. The numbers at branches indicate bootstrap results above 50%. Lines are drawn between the microsymbionts and their hosts. The color code indicates the place of origin of the leave or of the set when homogenous. The groups numbers 1 and 2 on the right are according to Yokoyama et al. [19].

**Figure 2:** Distribution of* Coriaria* species. Root nodules have been sampled from* C. myrtifolia*,* C. arborea*,* C. nepalensis*,* C. japonica,* and* C. microphylla *growing in Mediterranean areas (Morocco and France), New Zealand, Pakistan, Japan, and Mexico, respectively. Short arrows indicate sampling sites for this study while long arrows indicate possible routes of dispersal as discussed.

**Table 1:** List of *Coriaria* root nodules and sequences used in this study.

Species	Locality coordinates/altitude (asl)	Nodule labels	Plant sequence accession number		Bacterial sequence accession number			References
			ITS1-ITS2	*mat*K	*gln*A	*dna*A	IGS *nif*D-K	
*C. myrtifolia *	*Morocco *							
	Oued El Koub, Ouezzane: 35°01′879N/05°20′565E/140 m	CmMs1	KC796592	KC796601	KC796522	KC796582	KC796555	This study
		CmMs2 CmMs3 CmMs4			KC796523 KC796524 KC796525	KC796583 KC796584 KC796585	KC796556 KC796557 KC796558	This study This study This study
	Bab Berred, Chefchaouen: 35°00′979N/04°58′092′′E/1290 m	CmM1a	KC796590	KC796599	KC796517	KC796578	KC796550	This study
		CmM1b			KC796518	KC796579	KC796551	This study
		CmM1c			KC796519	KC796580	KC796552	This study
		CmM2a	KC796591	KC796600	KC796520	—	KC796553	This study
		CmM2b			KC796521	KC796581	KC796554	This study
	*France *							
	Nyons, 44°21′46.50′′N/5°08′21.82′′E/259 m	CmNy1	KC796598	KC796603	KC796531	KC796591	KC796564	This study
		CmNy2 CmNy3 CmNy4 CmNy5			KC796532 KC796533 KC796534 KC796535	KC796592 KC796593 KC796594 KC796595	KC796565 — KC796566 KC796567	This study This study This study This study
	Montpellier, 43°36′51.48′′N/3°52′23.97′′E/41 m	CmF1			KC796526	KC796586	KC796559	This study
		CmF2	KC796593	KC796602	KC796527	KC796587	KC796560	This study
		CmF3 CmF4 CmF5			KC796528 KC796529 KC796530	KC796588 KC796589 KC796590	KC796561 KC796562 KC796563	This study This study This study
			AF280102					Yang et al., unpublished
				AB016459				(Yokoyama et al., 2000 [19])

*C. japonica *	*Japan *							
	Tosa district, +33°45′39.18′′, +133°27′42, 89′′/10 m	CjJA		KC796605	KC796536	KC796503	KC796576	This study
		CjJB	KC796594		KC796537	KC796504	KC796577	This study
		CjJC CjJD CjJE			KC796538 KC796539 KC796540	KC796505 KC796506 KC796507	KC796578 KC796579 KC796580	This study This study This study
			AF280101					Yang et al., unpublished
				AB016456				(Yokoyama et al., 2000 [19])

*C. nepalensis *	*Pakistan *							
	Murree, +33°54′15′′N 73°23′25′′E/33.9042°N 73.3903°E/2291.2 m	CnP1	KC796597	KC796607	KC796544	KC796508	KC796584	This study
		CnP2			KC796545	KC796509	KC796585	This study
		CnP3			KC796546	KC796510	KC796586	This study
		CnP4						
			AF280103					Yang et al., unpublished

*C. arborea *	*New Zealand *							
	Hapuku river, North Canterbury, South island: −42°23′42.24′′, +173°41′18.07′′/64 m	CaNZ1	KC796595	KC796604	KC796542	KC796511	KC796581	This study
		CaNZ2			KC796543	KC796512	KC796582	This study
		CaNZ3			KC796544	KC796513	KC796583	This study
				AB16454				(Yokoyama et al., 2000 [19])
			EF635457					Rotherham et al., unpublished
			EF635475					Rotherham et al., unpublished
			AF277293					Yang et al., unpublished

*C*. *microphylla *	*Mexico *							
	Morelos, 99°30′, 19°30′/2400 m	CmicMx1	KC796596	KC796606	KC796547	KC796514	KC796587	This study
		CmicMx2			KC796548	KC796515	KC796588	This study
		CmicMx3			KC796549	KC796516	KC796589	This study
			AY091813					Yang et al., unpublished
				AB016458				(Yokoyama et al., 2000 [19])

*C. intermedia *			AF280100					Yang et al., unpublished
				AB016455				(Yokoyama et al., 2000 [19])

*C. terminalis *			AY091817					Yang et al., unpublished

*C. ruscifolia *			AY091815					Yang et al., unpublished
			AY091814					Yang et al., unpublished
			AF280104					Yang et al., unpublished
				AB016462				(Yokoyama et al., 2000 [19])

*C. sarmentosa *			AY091816					Yang et al., unpublished
				AB016464				(Yokoyama et al., 2000 [19])

*C. papuana *				AB016461				(Yokoyama et al., 2000 [19])

*Datisca glomerata *					CP002801	CP002801	CP002801	(Persson et al., 2011 [50])
			AY968449					Zhang et al., unpublished
				AF485250				Forrest and Hollingsworth unpublished
					

*Casuarina equisetifolia *					CP000249	CP000249	CP000249	(Normand et al., 2007 [51])
				AB015462				Sogo et al., unpublished
			AY864057					Herbert et al., unpublished

**Table 2:** Primers used for PCR amplification and DNA sequencing.

Gene primers	Sequence (5′-3′)	Amplicons approximate size (bp)	References
*gln*A			
DB41	TTCTTCATCCACGACCCG	500	(Clawson et al., 2004 [4])
DB44	GGCTTCGGCATGAAGGT		
*dna*A			
F7154_dnaAF	GAGGARTTCACCAACGACTTCAT	700	Bautista et al. unpublished
F7155_dnaAR	CRGAAGTGCTGGCCGATCTT		
IGS *nif*D-K			
F9372_nifD1 5	GTCATGCTCGCCGTCGGNG	700	This study
F9374_nifK1 5	GTTCTTCTCCCGGTAyTCCCA		
F9373_nifD2 5	ACCGGCTACGAGTTCGCNCA	700	This study
F9375_nifK2 5	TGCGAGCCGTGCACCAGNG		
18S-ITS1-5.8S-ITS2-28S			
ITS1	TCCGTAGGTGAACCTGCGG	700	(White et al., 1990 [52])
ITS4	TCCTCCGCTTATTGATATGC		
F9030-CJ-ITSF	AGCCGGACCCGCGACGAGTTT	400	This study
F9031-CJ-ITSR	CGACGTTGCGTGACGACGCCCA		
*mat*K			
F9249-matKF	ACATTTAAATTATGTGTCAG	700	This study
F9250-matkR	TGCATATACGCACAAATC		
